RETRACTED

# Analysis of Helicobacter pylori's Antibiotic Resistance Rate and Research on Its Eradication Treatment Plan

**DOI:** 10.1155/2021/6009602

**Published:** 2021-12-03

**Authors:** Li Jiao, Junmin Wang, Huan Ma

**Affiliations:** Department of Gastroenterology, The Third Hospital of Hebei Medical University, Shijiazhuang 050000, China

## Abstract

How to choose the right plan is the key to treatment, and this must take into account the local eradication of Helicobacter pylori and the drug resistance of Helicobacter pylori. In order to better eradicate Helicobacter pylori, in the current clinical treatment process, most of the combined treatments of triple drugs are used, but the therapeutic effect is still not ideal. In addition, many studies have focused on changing the types and dosages of drugs, but they have not yet achieved good results. This paper combines experimental research to analyze the drug resistance rate of Helicobacter pylori and obtains gastric mucosal specimens of patients through gastroscopy to cultivate clinical isolates of H. pylori.. Furthermore, this study used the Kirby-Bauer drug susceptibility disc technique to determine the sensitivity of H. pylori clinical isolates to a range of regularly used clinical antibiotics, as well as a set of instances of H. pylori antibiotic resistance. Finally, this research integrates experimental analyses and various successful eradication treatment plans to provide a unique eradication treatment strategy.

## 1. Introduction

Helicobacter pylori (H. pylori) is a spiral-shaped, microaerobic gram-negative bacterium. Helicobacter pylori is a recognized pathogen of human chronic gastritis, peptic ulcer, and gastric mucosa-associated lymphoid tissue (MALT) lymphoma and is closely related to the occurrence of gastric cancer. There are many resistance mechanisms of H. pylori, and the main reasons are as follows. One is the mutation of the corresponding drug resistance gene, which can produce drug resistance by changing the drug-metabolizing enzymes or targeting to modify the drug action site and reduce the permeability of the cell membrane. The second is to actively pump intracellular drugs out of the cell through the efflux pump. Bacterial efflux pumps are a class of transporter systems that may expel hazardous substrates from bacteria. They can efflux a wide range of medicines and metabolites that are toxic to bacteria. It is a result of bacteria adjusting to their surroundings. Furthermore, efflux pumps are found everywhere in bacteria and have a broad range of substrates, and their expression is vital in a number of bacteria's primary and secondary drug resistance. The efflux pump mainly uses the following two ways to make bacteria resistant. One is to enable bacteria to survive successfully at a certain concentration of antibiotics through the function of efflux antibiotics. The second is to provide surviving bacteria with further opportunities for specific drug resistance (such as drug target mutations) [1]. The efflux pump system associated with bacterial drug resistance is mostly composed of the following five families [2]: (1) transporters of ATP-binding cassettes (ABC type), (2) superfamily of major facilitators (MFS type), (3) superfamily of drug/metabolite transporters (DMT type), (4) extrusion of many drugs and hazardous compounds (MATE category), (5) family of resistance-nodulation-division (RND category) [3]. Except for ABC, which is powered by ATP, and MATE, which trades medicines through Na+, the other three kinds of transporters are powered by proton driving force and act as antiporters for protons and pharmaceuticals. That is, during the transit of protons and pharmaceuticals, protons enter the cell while drugs are expelled outside, with the latter being the predominant kind in prokaryotes.

RETRACTED

There are several active efflux transporters for antibiotics. Among these, only Gram-negative bacteria have the RND efflux pump family. The AcrAB-TolC efflux pump is the primary cause of multidrug resistance in Gram-negative bacteria among the RNDs. Numerous Gram-negative bacteria, such as Acinetobacter baumannii and Escherichia coli, acquire drug resistance, particularly multidrug resistance, through the dominant efflux system. It is capable of reacting with a broad variety of substrates, including tetracycline, chloramphenicol, and erythromycin, as well as B-lactams, puromycin, rifampicin, fluoroquinolones, oxidants, organic solvents, and basic dyes. Three components comprise the AcrAB-TolC efflux system: AcrB, AcrA, and TolC. AcrB is an efflux pump protein in the AcrAB-TolC efflux system, commonly known as the inner membrane transporter, that may excrete a range of medicines using protons as a driving force. TolC is the outer membrane channel protein of the AcrAB-TolC efflux system, which is formed of three subunits; AcrA is the membrane fusion protein of the AcrAB-TolC efflux system, and its major purpose is to join AcrB and TolC to create a triad complex. Porin is a protein that stretches from the outer membrane to the periplasm. The extracellular end of TolC is an open structure to provide an open outlet for the substrate, while the intracellular end is closed in a cone shape, and part of the protein is in the form of *α*-helix. It enters the periplasm and combines with AcrA to induce changes in the coiled-coil structure at the bottom, thereby opening the bottom opening, allowing the substrate to smoothly enter the porin and be discharged. During the efflux process, AcrB captures harmful substances in the bacteria. When the substrate binds to it, TolC binds to AcrAB and opens its internal channel to pump harmful substances out of the bacteria.

RETRACTED

This paper combines experimental research to analyze the drug resistance rate of Helicobacter pylori and combines experimental analysis to propose a specific eradication treatment plan to provide a theoretical reference for the subsequent treatment of Helicobacter pylori.

## 2. Related Work

Literature [4] used the proton-dynamic uncoupling agent carbonylcyanide-m-chlorophenylhydrazone (CCCP) to treat the ARHp80 strain without gene knockout. It is found that the rate and level of ethidium bromide accumulation in the ARHp80 strain treated with CCCP were significantly higher than that in the untreated ARHp80 strain. It is confirmed that H. pylori, like other Gram-negative bacteria, has an efflux pump that causes multidrug resistance and may play a role in antibiotic resistance. Literature [5] showed that the AcrAB-TolC efflux pump is involved in the resistance of H. pylori to metronidazole and clarithromycin. Literature [6] employed insertion mutation to simultaneously knock out a single or two genes producing outer membrane channel proteins (hefA and hefD) in the metronidazole-resistant strain H. pylori l061 generated in vitro. Additionally, it used gene sequencing to rule out the influence of mutations in the metronidazole-specific resistance genes rdxA and frxA on drug resistance. It is proven that the AcrAB-TolC efflux pump is involved in the metronidazole resistance of Helicobacter pylori. Literature [7] revealed that metronidazole-resistant Helicobacter pylori strains displayed high levels of hefA and hefD, which increased in response to metronidazole exposure. Additionally, metronidazole expression rises as the concentration of metronidazole increases, suggesting that metronidazole might produce high levels of the AcrAB-TolC efflux system, resulting in drug resistance. Additionally, literature [8] revealed that H. pylori strains that are susceptible to metronidazole may generate drug resistance when exposed to low doses of metronidazole while overexpressing hefA. Additionally, all of this happened prior to the reduction in metronidazole nitroreductase activity, implying that overexpression of the AcrAB-TolC efflux system is the first stage in the establishment of metronidazole resistance. Literature [9] shows that the AcrAB-TolC efflux pump was enhanced in 15 H. pylori strains resistant to clarithromycin. Clarithromycin's MIC for Helicobacter pylori dropped after treatment with the efflux pump inhibitor phenyl-arginine-naphthylamide (PAN), and it was concentration-dependent with PAN. It demonstrates that the AcrAB-TolC efflux pump also plays a critical role in H. pylori resistance to clarithromycin. Recently, researchers have identified the influence of the AcrAB-TolC efflux pump on H. pylori multidrug resistance using an in vitro produced H. pylori MDR strain. Literature [10] examined the H. pylori MDR strain produced by chloramphenicol and discovered an increase in the expression of hefA, the efflux pump's AcrAB-TolC efflux pump. Additionally, silencing the hefA gene or administering CCCP and proton pump inhibitors may drastically lower the MIC of a range of antibiotics against H. pylori MDR strains. It is hypothesised that the hefA gene of the AcrAB-TolC efflux pump contributes to the development of H. pylori multidrug resistance and that inhibiting the efflux pump may reverse the resistance.

RETRACTED

At the moment, research on the bacterial efflux pump is mostly focused on Escherichia coli and Acinetobacter baumannii, with little emphasis on Helicobacter pylori. Additionally, H. pylori research is mostly focused on experimentally created H. pylori resistance strains in vitro, most notably multidrug resistant strains induced by chloramphenicol. The resistance mechanisms of these strains and natural MDR strains isolated from clinical patients are not identical, and the study's findings may not be applicable to clinical H. pylori eradication therapy [11]. Simultaneously, the majority of studies examining the expression of genes producing H. pylori efflux pump-related proteins have identified just a subset of these genes and have not revealed alterations in the relevant antibiotic resistance genes. The AcrAB-TolC efflux pump-related protein coding genes are not fixed and joined to create an efflux pump system, according to studies on other Gram-negative bacteria, although cross-matching is possible [12]. As a result, just recognizing a portion of the genes producing the AcrAB-TolC efflux pump-related protein does not provide a comprehensive picture of the AcrAB-TolC efflux pump. Changes in the expression and function of the efflux pump in bacteria, including E. coli, Salmonella, Pseudomonas aeruginosa, Campylobacter jejuni, and alterations in drug-specific target genes, have all been linked to bacterial resistance in recent research. [13]. In particular, the RND efflux pump plays an important role in the acquisition of “self-mutation and acquired” resistance of Gram-negative bacteria [14]. Therefore, to deeply understand the role and mechanism of the efflux pump in H. pylori resistance, it is necessary to observe the expression of the efflux pump gene in H. pylori-resistant strains and the mutation of the corresponding antibiotic resistance gene.

RETRACTED

Fluoroquinolone triple therapy is the use of PPI+amoxicillin+levofloxacin. Fluoroquinolone antibiotics are a class of broad-spectrum antibiotics, which are widely used in medicine and aquaculture. This regimen is recommended as the second-line treatment regimen after the first treatment fails. PPI is mainly metabolized in the liver by CYP2C19 in the cytochrome P450 (CYP450) family. Different CYP2C19 genotypes in the population will cause the same PPI to have different metabolic effects in different patients, and it is divided into slow-metabolized, fast-metabolized, and intermediate [15]. It has been reported in the literature that fluoroquinolone antibiotics can reduce the biotransformation process regulated by CYP2C19 through competitive inhibition, which can reduce the difference in the efficacy of PPI caused by different CYP2C19 genotypes, and has a synergistic effect with PPI drugs [16]. However, levofloxacin also has a high resistance rate. Some studies use moxifloxacin instead of levofloxacin. Studies have found that when lansoprazole or omeprazole is used in triple therapy containing clarithromycin, the efficacy of PPI is affected by CYP2C19 gene polymorphism. However, there was no significant effect when using rabeprazole or esomeprazole [17]. Rabeprazole may be related to its nonenzymatic metabolism and is not affected by CYP2C19 gene polymorphism. Esomeprazole may be related to its pure S-isomer, but the specific mechanism is not clear, and there is currently no consensus on the optimal PPI selection [18]. The triple therapy of rifampicin is PPI+amoxicillin+rifampin. As a conventional antituberculosis drug, rifampicin is not often selected as a treatment for Helicobacter pylori infection, considering its adverse effects. Moreover, more and more clinical trials have confirmed that the regimen containing rifampicin actually has a good therapeutic effect on Helicobacter pylori infection [19]. Under the premise of no drug susceptibility test, the Toronto consensus on the treatment of adult Helicobacter pylori infection lists it as the only fourth-line treatment [20].

## 3. Experimental Method

The study subjects were patients having gastroscopy. Stomach mucosa tissues from the gastric antrum 2-3 cm from the pylorus were obtained as specimens under the gastroscope with the agreement of the patients based on particular inclusion and exclusion criteria. After obtaining permission, we utilised biopsy forceps to bite a piece of gastric mucosal tissue 2-3 cm from the pylorus in the stomach antrum. We rapidly transfer the specimen into an EP tube filled with Brinell broth and seal it using a disposable sterile needle (wipe the EP tube with alcohol before opening and closing the EP tube). All specimens must be submerged in liquid and sealed off from the environment. We put the EP tube vertically into a foam box filled with ice cubes and labelled the specimen with the following basic information: name, gender, age, major complaint, microscopic diagnosis, prior medication history, collection date, and hospitalisation numbers for inpatients.

RETRACTED

Within four hours, gastric mucosal specimens must be infected. We removed the H. pylori separation medium from the refrigerator and put it at room temperature. In the biological safety cabinet, we take up the specimen with a disposable sterile needle, and the mucosal surface comes into touch with the culture media. Following that, utilising the cryopreserving gradient one-way smear inoculation approach, we employ a sterile inoculation loop to completely spread the specimens on the culture medium (Zigzag streak method). Following that, we inverted the injected H. pylori separation medium in a clear airtight culture tank, added a microaerobic gas bag and a little quantity of sterile water, and placed it in a constant temperature shaker set at 37°C for 3-7 days.

We removed the H. pylori culture media from the refrigerator and deposited it at room temperature. In the biological safety cabinet, we employ a sterile inoculating loop to select colonies recognised as clinical isolates of Helicobacter pylori and inoculate them using the dense 3-zone streaking technique on the H. pylori subculture medium. In a clear airtight culture tank, we placed the infected H. pylori subculture medium upside down, added a microaerobic gas bag and a little quantity of sterile water, and placed it in a constant temperature shaker set to 37°C for 3-7 days.

We took out the H. pylori drug-sensitive medium and placed it at room temperature. We used disposable sterile cotton swabs to pick out pure colonies in the biological safety cabinet and mixed them in sterile normal saline to generate a homogeneous bacterial solution. The concentration of the bacterial solution is 1.5 × 10^8^ cfu/ml, which is equivalent to the turbidity of No. 0.5 McDonald's turbidity tube. We replaced a cotton swab soaked in the bacterial suspension, squeezed the excess liquid on the tube wall, and smeared it evenly in 3 different directions 3 times to form a uniform inoculation layer on the drug sensitive medium. After the medium dries a little, a Kirby-Bauer drug susceptibility paper will be affixed within 15 minutes according to the requirements of the drug susceptibility test. We used a sterile filter paper sheet of the same size and thickness as the drug sensitive paper sheet as a blank control group and placed it in a constant temperature shaker at 37°C for 3-7 days. After taking it out, we observe whether there is an obvious zone of inhibition in the culture medium, measure and record the diameter of the zone of inhibition with a vernier caliper, and read and record the result according to the instructions of the drug-sensitive paper manufacturer.

RETRACTED

To confirm the sensitivity of H. pylori to antibiotics, a drug sensitivity test was performed again. The E-test method was used to detect the MIC of 8 antibiotics (AM, MZ, CH, LE, TC, MX, RI, and AZ) against H. pylori. The E-test method is an intuitive and direct quantitative technique that combines the principles of diffusion and dilution methods for bacterial susceptibility testing. There is a preprepared antibiotic on the back of the test strip, and its concentration increases continuously and exponentially. The front side is marked with the specific value of MIC, the unit is *μ*g/ml, and the value can be read intuitively. According to the National Committee for Clinical Laboratory Standards (NCCLS) standards, the bacteria are judged as resistant or sensitive. MIC ≥ 1 *μ*g/ml is defined as amoxicillin resistance, MIC ≥ 8 *μ*g/ml is defined as metronidazole resistance, MIC ≥ 1 *μ*g/ml is defined as clarithromycin resistance, and MIC ≥ 1 *μ*g/ml is defined as levofloxacin resistance. MIC ≥ 1 *μ*g/ml is defined as tetracycline resistance, MIC ≥ 1 *μ*g/ml is defined as moxifloxacin resistance, MIC ≥ 1 *μ*g/ml is defined as rifampicin resistance, and MIC ≥ 1 *μ*g/ml is defined as azithromycin resistance. The drug susceptibility test was performed with the standard strain HP11637 at the same time as the quality control, and the drug susceptibility test was repeated 3 times. The specific operation method is carried out in accordance with the standardized operation process of clinical laboratories in the United States, and the experimental steps are as follows. (1) We use a sterile inoculating loop to scrape H. pylori in the logarithmic growth phase into an EP tube containing 1 ml of sterile physiological saline. (2) We use a turbidimetric meter to adjust the concentration of the bacterial solution to 2.0 McDonnell's concentration. (3) We use a pipette to pipette about 1 ml of the adjusted concentration of the bacteria liquid onto the sterilized small plastic cup. (4) We use a spiral spreader to suck 200 *μ*l of bacteria in the plastic cup and spread it evenly on a Muller-Hinton (MH) agar medium plate with a diameter of 150 mm. (5) We place the agar plate for a few minutes and let it dry naturally. (6) We use sterile tweezers to attach the E-test test strip to the surface of the agar medium. (7) We place it in a three-gas incubator and culture it for 48-72 h in a microaerobic environment. (8) The agar plate was removed for observation, and the MIC of each antibiotic against the bacterium was determined. The MIC is the scale at the intersection of the oval antibacterial ring and the test strip. The strain is classified as either sensitive or resistant by the National Committee for Clinical Laboratory Standards (NCCLS).

RETRACTED

We use the K-B method to detect the sensitivity of H. pylori to furazolidone (FR). The K-B method is to stick a filter paper sheet containing a quantitative antimicrobial drug on the surface of agar that has been inoculated with the test bacteria, and the drug in the sheet of paper diffuses in the agar. As the diffusion distance increases, the concentration of antibacterial drugs decreases logarithmically, thereby forming a concentration gradient around the paper. While the drug spreads, the test bacteria within the inhibitory concentration range around the paper cannot grow, while the strains outside the inhibitory concentration range continue to grow, thereby forming a transparent bacteriostatic zone around the paper. Because of the impact of the drug's diffusion rate in the agar, the width of the inhibition zone of various antibacterial agents may vary. The extent of the zone of inhibition might represent the tested bacteria's sensitivity to the tested drug and is inversely connected with the drug's minimum inhibitory concentration (MIC) for the tested bacterium. That is, the lower the MIC, the bigger the inhibition zone. The mm unit is used to interpret the zone of inhibition. The bacteria are classified as resistant or sensitive according to the National Committee on Clinical Laboratory Standards (NCCLS). The diameter of the inhibition zone ≤ 7 mm is considered to be furazolidone resistance. The drug susceptibility test is performed with the standard strain HP11637 at the same time as the quality control. The specific operation method is carried out in accordance with the standardized operation process of clinical laboratories in the United States, and finally, the results are interpreted, the diameter of the inhibition zone is measured with a caliper, and then, the reading is performed, and the drug susceptibility test is repeated 3 times.

## 4. Result

This paper shows the disease distribution of the isolated strains obtained through experimental statistics in Table 1 and Figure 1.

The susceptibility test findings of clinical isolates of H. pylori to eight medications, including metronidazole, levofloxacin, clarithromycin, amoxicillin, moxifloxacin, furazolidone, tetracycline, and rifampin, are examined in this research. The drug resistance is counted, and the results are shown in Tables 2–9.

RETRACTED

From the above analysis, it can be seen that the clinical isolates of H. pylori are resistant to metronidazole, levofloxacin, and clarithromycin. However, its resistance to amoxicillin, moxifloxacin, furazolidone, tetracycline, and rifampicin is low. It may be used as a guide during clinical treatment. For example, the resistance rate of H. pylori clinical isolates to metronidazole can be assumed to be 100%, and the inaccuracy can be attributed to strain contamination. The resistance rate of H. pylori clinical isolates to amoxicillin, moxifloxacin, furazolidone, tetracycline, and rifampicin may be assumed to be zero, and the inaccuracy can be attributed to strain contamination. H. pylori has harsh requirements for the growth environment, and it is still difficult to routinely culture in vitro in terms of current technology. The reliability, operational safety, and economic benefits of drug sensitivity experiments that are routinely used in clinical practice are still to be studied. As a result, we may employ empirical therapy for newly treated patients based on recommendations, prior medication history, and known knowledge on antibiotic resistance in the area to ensure that antibiotics are given in combination, in suitable quantities, and throughout the complete course of treatment. There are grounds for radical therapy in individuals with resistant H. pylori infection who have failed the first treatment, failed the second treatment, or failed three or more treatments. Within the scope of the patient's economic and psychological tolerance, radical treatment is recommended based on the results of drug sensitivity experiments.

## 5. Conclusion

Future areas for research to increase the success rate of clinical H. pylori infections include the following: (1) It is vital to monitor patients having radical surgery, document their prior medication history, the treatment plan followed at the time, and the outcome of the procedure. (2) It is required to conduct large-scale clinical studies on a regular basis to target the population and confirm resistance to H. pylori antibiotics in the region. (3) Vaccine research and development must be maintained. (4) It is important to create a safe, low-cost, high-efficiency, reliable, simple, and rapid approach for evaluating H. pylori resistance on a broad scale. Unlike the conventional approach of culturing Helicobacter pylori from the stomach mucosa and then conducting the medication susceptibility test, this method may be integrated with developing gene detection technologies. There have been a large number of studies on the mechanism of H. pylori gene mutations leading to drug resistance, and there have been many clinical research reports using PCR gene chips in the detection of H. pylori infection, the genotype of PPI metabolic enzymes and the acquisition of drug resistance information. The latest MaastrichtV consensus recommendation can be based on genetic testing results of H. pylori resistance to individualized antibiotic treatment. It is believed that the detection of H. pylori infection and the study of drug resistance are combined with chip technology to be the direction of future development.

RETRACTED

## Figures and Tables

**Figure 1:** Histogram of disease distribution of isolated strains.

**Table 1:** Statistical table of disease distribution of isolated strains.

Disease	Proportion (%)
Gastric proliferative lesions	27.51%
Duodenal ulcer	27.51%
Stomach ulcer	12%
Compound ulcer	12%
Chronic superficial gastritis	18%
Chronic atrophic gastritis	12%

**Table 2:** The resistance of H. pylori to metronidazole.

No.	Resistance rate (%)	No.	Resistance rate (%)	No.	Resistance rate (%)
1	99.636	16	99.525	31	99.894
2	99.679	17	99.881	32	99.237
3	99.275	18	99.837	33	99.272
4	99.427	19	99.955	34	99.956
5	99.316	20	99.850	35	99.507
6	99.286	21	99.717	36	99.449
7	99.892	22	99.593	37	99.299
8	99.417	23	99.323	38	99.967
9	99.492	24	99.498	39	99.497
10	99.425	25	99.962	40	99.514
11	99.594	26	99.889	41	99.619
12	99.481	27	99.973	42	99.819
13	99.734	28	99.675	43	99.281
14	99.934	29	99.791	44	99.822
15	99.607	30	99.705	45	99.322

**Table 3:** Resistance of H. pylori to levofloxacin.

No.	Resistance rate (%)	No.	Resistance rate (%)	No.	Resistance rate (%)
1	22.016	16	23.045	31	22.700
2	23.846	17	22.775	32	23.187
3	22.021	18	23.252	33	22.005
4	22.387	19	22.985	34	23.884
5	23.116	20	23.160	35	22.668
6	22.833	21	23.271	36	23.951
7	22.927	22	22.613	37	23.615
8	22.337	23	22.868	38	22.593
9	23.102	24	23.422	39	22.869
10	23.614	25	23.810	40	23.716
11	23.099	26	22.616	41	22.857
12	22.161	27	23.216	42	22.856
13	23.844	28	23.391	43	22.281
14	23.231	29	22.315	44	22.478
15	23.777	30	23.225	45	23.025

**Table 4:** Resistance of H. pylori to clarithromycin.

No.	Resistance rate (%)	No.	Resistance rate (%)	No.	Resistance rate (%)
1	16.754	16	16.334	31	16.668
2	16.914	17	17.402	32	16.005
3	16.814	18	16.208	33	17.388
4	16.841	19	17.967	34	16.236
5	16.237	20	16.019	35	16.670
6	17.814	21	16.509	36	17.853
7	17.222	22	17.407	37	17.707
8	16.719	23	16.952	38	16.199
9	17.832	24	17.421	39	17.683
10	17.985	25	17.057	40	17.138
11	16.069	26	16.655	41	17.407
12	17.307	27	17.806	42	16.388
13	17.607	28	17.671	43	16.440
14	17.988	29	17.777	44	17.423
15	16.605	30	16.106	45	17.493

RETRACTED

**Table 5:** Resistance of H. pylori to amoxicillin.

No.	Resistance rate (%)	No.	Resistance rate (%)	No.	Resistance rate (%)
1	0.082	16	0.057	31	0.050
2	0.078	17	0.089	32	0.098
3	0.067	18	0.055	33	0.081
4	0.054	19	0.073	34	0.079
5	0.057	20	0.064	35	0.086
6	0.065	21	0.098	36	0.050
7	0.052	22	0.096	37	0.057
8	0.076	23	0.078	38	0.074
9	0.071	24	0.057	39	0.100
10	0.071	25	0.058	40	0.066
11	0.052	26	0.053	41	0.082
12	0.093	27	0.065	42	0.057
13	0.091	28	0.070	43	0.051
14	0.078	29	0.072	44	0.097
15	0.085	30	0.059	45	0.063

**Table 6:** Resistance of H. pylori to moxifloxacin.

No.	Resistance rate (%)	No.	Resistance rate (%)	No.	Resistance rate (%)
1	0.081	16	0.084	31	0.069
2	0.075	17	0.082	32	0.082
3	0.063	18	0.059	33	0.076
4	0.053	19	0.100	34	0.087
5	0.053	20	0.099	35	0.091
6	0.091	21	0.076	36	0.053
7	0.072	22	0.080	37	0.081
8	0.088	23	0.068	38	0.065
9	0.076	24	0.099	39	0.056
10	0.080	25	0.094	40	0.074
11	0.054	26	0.056	41	0.093
12	0.065	27	0.079	42	0.074
13	0.081	28	0.095	43	0.060
14	0.100	29	0.076	44	0.057
15	0.067	30	0.056	45	0.059

**Table 7:** Resistance of H. pylori to furazolidone.

No.	Resistance rate (%)	No.	Resistance rate (%)	No.	Resistance rate (%)
1	0.094	16	0.073	31	0.054
2	0.095	17	0.065	32	0.051
3	0.076	18	0.051	33	0.060
4	0.058	19	0.069	34	0.072
5	0.056	20	0.097	35	0.083
6	0.078	21	0.058	36	0.052
7	0.072	22	0.060	37	0.052
8	0.080	23	0.051	38	0.087
9	0.098	24	0.096	39	0.090
10	0.098	25	0.100	40	0.092
11	0.083	26	0.058	41	0.057
12	0.056	27	0.074	42	0.055
13	0.069	28	0.078	43	0.089
14	0.081	29	0.051	44	0.100
15	0.062	30	0.065	45	0.086

**Table 8:** Resistance of H. pylori to tetracycline.

No.	Resistance rate (%)	No.	Resistance rate (%)	No.	Resistance rate (%)
1	0.091	16	0.080	31	0.088
2	0.053	17	0.091	32	0.057
3	0.064	18	0.094	33	0.098
4	0.087	19	0.094	34	0.072
5	0.096	20	0.092	35	0.086
6	0.065	21	0.057	36	0.054
7	0.065	22	0.087	37	0.050
8	0.057	23	0.055	38	0.071
9	0.063	24	0.066	39	0.061
10	0.096	25	0.055	40	0.087
11	0.090	26	0.062	41	0.077
12	0.067	27	0.091	42	0.062
13	0.077	28	0.074	43	0.059
14	0.098	29	0.086	44	0.057
15	0.063	30	0.082	45	0.078

**Table 9:** Resistance of H. pylori to Merifampicin.

No.	Resistance rate (%)	No.	Resistance rate (%)	No.	Resistance rate (%)
1	0.063	16	0.071	31	0.091
2	0.062	17	0.051	32	0.054
3	0.099	18	0.065	33	0.066
4	0.061	19	0.055	34	0.061
5	0.088	20	0.064	35	0.082
6	0.051	21	0.080	36	0.084
7	0.089	22	0.061	37	0.080
8	0.070	23	0.054	38	0.097
9	0.083	24	0.066	39	0.087
10	0.079	25	0.100	40	0.059
11	0.063	26	0.093	41	0.069
12	0.085	27	0.081	42	0.078
13	0.094	28	0.080	43	0.093
14	0.053	29	0.052	44	0.078
15	0.092	30	0.099	45	0.060

## Data Availability

The data used to support the findings of this study are included within the article.
